# Edge-Aware Graph Neural Network for Multi-Hop Path Reasoning over Knowledge Base

**DOI:** 10.1155/2022/4734179

**Published:** 2022-10-12

**Authors:** Yanan Zhang, Li Jin, Xiaoyu Li, Honqi Wang

**Affiliations:** ^1^Aerospace Information Research Institute, Chinese Academy of Sciences, Beijing 100190, China; ^2^Key Laboratory of Network Information System Technology (NIST), Aerospace Information Research Institute, Chinese Academy of Sciences, Beijing 100190, China; ^3^University of Chinese Academy of Sciences, Beijing 100049, China; ^4^School of Electronic, Electrical and Communication Engineering, University of Chinese Academy of Sciences, Beijing 100190, China

## Abstract

Multi-hop path reasoning over knowledge base aims at finding answer entities for an input question by walking along a path of triples from graph structure data, which is a crucial branch in the knowledge base question answering (KBQA) research field. Previous studies rely on deep neural networks to simulate the way humans solve multi-hop questions, which do not consider the latent relation information contained in connected edges, and lack of measuring the correlation between specific relations and the input question. To address these challenges, we propose an edge-aware graph neural network for multi-hop path reasoning task. First, a query node is directly added to the candidate subgraph retrieved from the knowledge base, which constructs what we term a query graph. This graph construction strategy makes it possible to enhance the information flow between the question and the nodes for the subsequent message passing steps. Second, question-related information contained in the relations is added to the entity node representations during graph updating; meanwhile, the relation representations are updated. Finally, the attention mechanism is used to weight the contribution from neighbor nodes so that only the information of neighbor nodes related to the query can be injected into new node representations. Experimental results on MetaQA and PathQuestion-Large (PQL) benchmarks demonstrate that the proposed model achieves higher Hit@1 and F1 scores than the baseline methods by a large margin. Moreover, ablation studies show that both the graph construction and the graph update algorithm contribute to performance improvement.

## 1. Introduction

Knowledge base question answering (KBQA) is a task to figure out the entities as answers for an input question from a given knowledge base (KB) and has attracted many researchers to work on it [1–10]. It is a challenging academic task, especially when answering multi-hop questions. As shown in Figure 1, a 3-hop complex question example is given. The topic entity of the question, *“What languages are the movies that share directors with Dick Tracy in?”*, is *Dick Tracy*, and the multi-hop triplet path \{*(Dick Tracy, directed_by, Warren Beatty), (Warren Beatty, directed, Reds), (Reds, in_language, Russian)*\} needs to be extracted from the KB to find the answer *Russian*. Since the intermediate entity in multi-hop path reasoning is not unique, there may be multiple correct answers to the input question. For example, if the green node *Heaven Can Wait* in Figure 1 has the relation *in_language* with the entity *English*, the question will have two answers, *English* and *Russian*. Both precision and recall metrics are important for this type of multi-hop questions.

Early studies on multi-hop questions mainly focus on methods based on semantic parsing [11]. The intuitive idea is to convert a question into the corresponding structured query (e.g., in SPARQL) to extract the resulting entity from a KB. Although these methods prove effectiveness, their processing steps and conversion process are relatively complex and meanwhile may involve expert knowledge or heuristic rules. Considering that answering multi-hop questions requires searching for reasoning paths, starting from the entity mentioned in question, and consisting of both the relations at each hop and intermediate entities, recent studies [12–14] have focused on the power of graph neural networks (GNNs) to solve the above limitations. They often model the question directly to get a candidate entity graph, and then leverage graph neural network-based information propagation methods to update the node representations in the graph, which are used to choose the answer entities. However, the current GNN-based methods and multi-hop path reasoning over knowledge base tasks are not compatible enough.

For answering a multi-hop question, people usually start from the topic entity mentioned in the question and search for the corresponding relation path in turn until the answer entity to the question is reached. Because GNN retains a state that can represent information from its neighborhood with arbitrary depth, the GNN-based information propagation process can simulate this kind of human problem-solving idea. In one hop message passing, the information of neighboring nodes is passed to the current node. After multiple propagation, nodes outside of multiple hops will obtain the information of the reasoning path starting from the topic entity. If this path and the question are highly matched, the possibility that this node refers to the answer is very high. Based on this assumption, we believe that the node representation after message passing contains the pivotal information needed to answer the question. Therefore, improvements are made on the basis of GNN network to adapt it to the multi-hop path reasoning over knowledge base task. First, the information contained in the predicate is essential, which determines the degree of matching with the question. However, previous GNN-based models [14–16] mostly consider how to propagate information between entities, while predicate information is more used as the weight of entity information in the propagation, ignoring their semantic information. To solve the above issues, the predicate information on the edges of the graph needs to be used reasonably and the predicate representation needs to be updated during message passing. Second, the way that the question is updated is also essential, which relates to the interactive information with the candidate entity graph. The previous methods [2, 12–14] either fix the question representation or update it with the representation of all nodes in the graph. To solve the issues, further increasing the information interaction between the question and the entity nodes, improvements are made on the way to construct the graph. The question text is added to the entity graph as a node. Because the question contains the mention of the topic entity, the question node is directly connected to the topic entity node in the graph. In this way, during the graph update process, not only the information contained in the question is fused into the entity node representation but also the question node representation is also updated. To confirm the observations, we conducted experiments with our proposed model on two datasets, MetaQA [17] and PathQuestion-Large (PQL) [18], and the experimental results reached the state-of-the-art level. In particular, the F1 score has been significantly improved (the F1 score of our model is 10.7% and 28.6% higher than baselines on the MetaQA 2-Hop and 3-Hop, respectively), which shows that the proposed method improves Hit@1 without sacrificing the recall.

The main contributions of our paper can be summarized as follows: 1) We propose an edge-aware graph neural network to simultaneously update the representation of both the nodes and the predicate edges, better measuring the relevance of the question and relations for multi-hop path reasoning. 2) We construct a query graph, treat the question as a node, and connect it to the topic entity, which allows the question information to flow to candidate entities along the propagation path during updating the graph. 3) We conduct experiments on two widely used multi-hop KBQA datasets, MetaQA and PQL, to prove our theory and effectiveness of the proposed model.

## 2. Related Work

Multi-hop path reasoning over knowledge base aims at finding answer entities for an input question by walking along a path of triples from graph structure data, which is directly related to the existing KBQA research field. Besides, the method presented in our paper is similar to previous studies using GNN for question answering.

### 2.1. Knowledge Base Question Answering

Embedding based KBQA models are mainly divided into a single-hop task and multi-hop task. The single-hop KBQA models [19–23] predict the answer by judging the similarity between the question and relations in candidate triples. For example, Zhao et al. [20] proposed a joint scoring conventional neural network model that leverages subject-predicate dependency. Moreover, they used a novel well-order loss function to consider the different subject and predicate contributions to answer prediction. Zhou et al. [21] proposed a parameter-shared deep fused model that integrates subject detection and question-predicate matching in a unified framework. Wang et al. [23] used a multi-task learning framework to train a unified model, which shared a BERT encoder across all KBQA sub-tasks and define task-specific layers on top of the shared layer to reduce the cost.

Multi-hop KBQA tasks often adopt methods based on memory networks [24, 25], semantic parsing [26–28], or reinforcement learning [29–32]. For example, Xu et al. [25] improved traditional key-value memory networks to answer complex questions by designing a new query updating strategy to mask previously addressed memory information from the query representations, and they introduced a novel STOP strategy to read a flexible number of triples from memory slots. Maheshwari et al. [27] treated question answering as a problem of semantic query graph generation and re-ranking. They proposed a self-attention based slot matching model that exploits the inherent structure of the query graphs to learn how to rank core chain candidates. Hua et al. [31] took a meta-reinforcement learning approach to adapt the meta-learned programmer to new questions based on the most similar questions retrieved. To effectively create the support sets, they proposed an unsupervised retriever to find the questions that are structurally and semantically similar to the new questions from the training dataset. In addition, there are some other KBQA methods [33, 34]. For example, He et al. [34] proposed a novel teacher-student approach, in which the student network aimed to find the correct answer to the query, while the teacher network tried to learn intermediate supervision signals for improving the reasoning capacity of the student network. However, these methods lack of considering graph structure information contained in the KB. Recent studies [2, 13, 14] have introduced graph neural networks into multi-hop KBQA tasks, which is an efficient way to leverage graph structure information to represent complex relationships among entities. GNN-based methods will be introduced in detail in the following section.

### 2.2. Graph Neural Network Based Question Answering

Recent studies on multi-hop question answering attempt to build graphs based on entities and conduct reasoning over the constructed graph using graph neural networks [35–38], which are introduced to modify propagation limitation in long-distance relation. GNN-based question answering consists of many popular research directions, including reading comprehension, multiple-choice question answering, open domain question answering, and KBQA.

#### 2.2.1. Multi-Hop Reading Comprehension

GNN-based multi-hop reading comprehension approaches aggregate scattered pieces of evidence across documents into a graph and then employ GNN-based message passing algorithms to perform multi-step reasoning. This work proposed by [39] is the first attempt to explore how GNN can work in the context of multi-document reading comprehension. They constructed an entity graph, where nodes are entity mentions from supporting documents and edges encode relations between different mentions (e.g., within- and cross-document coreference), and then adapted a graph convolutional network (GCN) to answer questions by updating node representations based on neighborhood features. The subsequent research work based on GNN can be roughly divided into two directions. One direction is to calculate the graph node representation [40–42]. For example, Cao et al. [40] applied bi-directional attention between an entity graph and input query after GCN reasoning over the graph to formulate a query-aware node representation, which could derive the mutual information between the query and entities for final prediction. Tang et al. [41] proposed a Gated-RGCN to utilize the attention and question-aware gating mechanism to regulate the usefulness of information propagating across documents and add question information during reasoning. The other direction is the graph construction [43–46]. For example, Tu et al. [43] constructed a heterogeneous graph, which contained different types of nodes (not just entity nodes) representing different granularity levels of information. Fang et al. [44] constructed a hierarchical graph to connect clues from different sources.

#### 2.2.2. Question Answering over Knowledge Base

The research direction, commonsense question answering [15, 16], also uses the external KB as one information source to answer questions. For example, Feng et al. [16] equipped pre-trained language models with a multi-hop graph relation network, which inherits the interpretability of path-based models and the scalability of GNNs. Yasunaga et al. [15] designed a joint graph and proposed the node relevance scoring function to estimate the importance of KB nodes related to the question context. However, commonsense question answering, also called multiple-choice question answering, only needs to choose one answer from a fixed number of candidate options, which is equivalent to a simplified version of the KBQA task where any entity in the KB may be the specified answer. Moreover, several work [12, 47, 48] studied question answering over the combination of a large-scale KB and entity-linked text task, called open domain question answering. For example, Sun et al. [12] proposed a novel heterogeneous update rule based on GCN to aggregate evidence across different information sources. And they proposed an integrated framework called PullNet in follow-up published work [48], which used an iterative process to construct a question-specific subgraph containing information relevant to the question. However, these models pay more attention to the problem of heterogeneous information fusion.

GNN-based KBQA approaches [2, 13, 14, 49] are most closely related to our method. The work proposed by [49] is the first attempt to apply GNNs to KBQA. They proposed to use the GNN to encode the graph structure of the semantic parse. Wang et al. [14] introduced a novel model based on GNNs to capture long-distance node information. Han et al. [2] proposed a directed hypergraph convolutional network to handle multi-hop KBQA task, which leverages hyperedges to connect more than two nodes more than pairwise connection. Moreover, they designed a dynamic relation strategy for dynamically updating relation states and paying attention to different relations at different hops during the reasoning process. Different from these models, our paper focuses on the message flow and the interaction between the query with the candidate graph. We not only construct a query graph to allow a two-way interaction of question information and candidate entity information but also design an edge-aware message passing algorithm for fusing relation information into the entity representation to facilitate the final matching of questions and candidates.

## 3. Task definition

Let *𝒦*={*𝒱*, *ℰ*, *ℛ*} denote a knowledge base, where *𝒱* is the set of entities, *ℛ* is the set of relations, and *ℰ* is the set of triples in the KB. A triple *t* ∈ *ℰ* is denoted as *t*=(*s*, *r*, *o*), where *s*, *o* ∈ *𝒱* are entities and *r* ∈ *ℛ* is the relation between head entity *s* and tail entity *o*. Given a multi-hop path question *Q*=(*w*_1_, *w*_2_,…, *w*_*n*_), where *w*_*j*_ denotes the *j*th word and *n* is the length of the question word sequence. The question contains only one topic entity *s*_1_ ∈ *𝒱*, which can be annotated by some existing entity linkers, and its answer can be found by walking down a triplet path {*t*_1_, *t*_2_,……, *t*_*L*_}⊆*ℰ*, where *t*_*l*_ denotes the *l*-hop triple answering the question *Q*. The first hop triple *t*_1_=(*s*_1_, *r*_1_, *o*_1_) starts from the topic entity of *Q*, and the last hop triple *t*_*L*_=(*s*_*L*_, *r*_*L*_, *o*_*L*_) ends with the answer entity. Note that *o*_*l*−1_ in (*l* − 1)-hop triple and *s*_*l*_ in *l*-hop triple are the same entity. The task is to find a triple path from *ℰ* and extract its end entity as the reasoning answer.

## 4. Method

As shown in Figure 2, to reason over a given query context using specific knowledge from a KB, the edge-aware GNN model consists of four main components. First, retrieve the subgraph *G*_*c*_ corresponding to the given question from the KB, and construct the query graph *G*_*q*_ by connecting the query node to the topic entities in *G*_*c*_. Second, encode the query graph *G*_*q*_, where nodes and edges are initialized as corresponding embeddings. Third, update the query graph *G*_*q*_ by using GNN-based information propagation for multiple rounds. Finally, predict the answer based on the relevance scores of both the final query node and candidate entity node representations. The details of each phase are described in the following sections.

### 4.1. Graph Construction

Given a question *Q*, the topic entity *s*_1_ can be identified by any entity linker. Then, a subgraph *G*_*c*_ can be retrieved from the KB by querying *N*-hop entities around the topic entity *s*_1_, which contains answer entities. All entity nodes in the subgraph are candidate entities {*C*_*q*_}. Traditional GNN-based methods directly perform message propagation on the retrieved subgraph *G*_*c*_. To strengthen information flowing between the question and entity nodes in the following information propagation, a new query node *q* representing the question context is introduced into the above subgraph, where *q* is connected to the topic entity *s*_1_ using a new predicate type *r*_*q*_. Note that the predicate type represents the relationship between the query context and the relevant entities in *G*_*c*_. Such a newly obtained graph containing the query and candidate nodes is termed as query graph *G*_*q*_.

### 4.2. Graph Encoder

The graph encoder layer initializes all graph nodes representing entities, and graph edges representing predicates to vector representation. The node embedding for *q* is initialized by using a long short-term memory network (LSTM) to encode the query context *e*_*q*_=*LSTM*(*w*_1_, *w*_2_,…, *w*_*n*_), where *e*_*q*_ ∈ *R*^*d*^ is the last state of LSTM output and *d* is the hidden state size. Specifically, a LSTM has several cell layers to make memories, and each cell layer involves the forget, input, and output gates. Let *f*_*j*_, *i*_*j*_, and *o*_*j*_ denote the *j*th cell layer outputs of forget, input, and output gates. The following formula elaborates the technical details of the *j*th cell layer:

(1) $$\begin{array}{c} f_{j}=\sigma \left(W_{f}w_{j}+V_{f}s_{j-1}+b_{f}\right)\text{,}\\ i_{j}=\sigma \left(W_{i}w_{j}+V_{i}s_{j-1}+b_{i}\right)\text{,}\\ o_{j}=\sigma \left(W_{o}w_{j}+V_{o}s_{j-1}+b_{o}\right)\text{,}\\ c_{j}=f_{j}⊗c_{j-1}+i_{j}⊗\tan\;h\left(W_{c}w_{j}+V_{c}h_{j-1}+b_{c}\right)\text{,}\\ s_{j}=o_{j}⊗\tan\;h\left(c_{j}\right)\text{,} \end{array}$$

where *c*_*j*_ is the cell state for long-term memory, *s*_*j*_ is the intermediate state for short-term memory, *W* and *V* with different subscripts are the weight matrices, and *b* with different subscripts is bias vectors. In addition, *σ*( ) is a Sigmoid function, tan *h*( ) is a Tanh function, and ⊗ denotes the element-wise multiplication. The value of intermediate state of the last cell layer, *s*_*n*_, is the query node embedding *e*_*q*_.

Other nodes and edges on *G*_*q*_ are initialized by using pre-trained word vectors or random initialized vectors. Let *e*_*m*_ represent the entity vector for entity node *m* in *G*_*c*_, and *x*_*r*_ represent the predicate vector for predicate edge *r* in *G*_*q*_. The nodes and edges in the graph are stored in the entity matrix *E*={*e*_1_,…, *e*_*n*_*e*__} and fact matrix *R*={*x*_1_,…, *x*_*n*_*r*__}, respectively, where *E* ∈ *R*^*n*_*e*_*∗d*^, *R* ∈ *R*^*n*_*r*_*∗d*^, *n*_*e*_ is the number of entity nodes in the graph *G*_*c*_, *n*_*r*_ is the number of triples in the graph *G*_*q*_, and *d* is the embedding size that is equal to the hidden state size of the LSTM.

### 4.3. Multi-Hop Graph Update

The basic recipe for graph-propagation based models is to update node representations via iterative message passing between neighbors on the graph. This phase is called message passing (namely, information propagation) that runs for *L* time steps (namely, *L* hops). The general formulas of node update are defined as follows:

(2) $$\begin{array}{c} h_{m}^{\left(l\right)}=\chi \left(h_{m}^{\left(l-1\right)},\underset{r}{\sum }\underset{k\in N_{r}\left(m\right)}{\sum }\psi \left(h_{k}^{\left(l-1\right)},x_{r}\right)\right)\text{,} \end{array}$$

where *l* ∈ {1,…, *L*} is the hop number, *N*_*r*_(*m*) denotes all the entity neighbors of the current node *m* along the incoming edges of relation *r*, *χ* is an updating function, and *ψ* represents a message function. In (2), the updating function and message function can be any reasonable model or algorithm, which can be designed according to different targets. These two function designed in our model will be described in detail in the following section.

During the graph updating process, our edge-aware GNN model has conducted three strategies to enhance the path reasoning performance. First, every time node representations are updated, only if the information of neighbor nodes related to the query is calculated. Second, in order to get the node representations matching the input query, the edge information needs to be incorporated once the node is updated. Third, since relation information and query information are equally important, in addition to entity node representations, both query node and edge representations also need to be updated once an update operation is triggered. In conclusion, every time the graph is updated, there are three aspects that need to be updated: the relation edges *R*, the entity nodes *E*, and the query node *e*_*q*_ in the graph *G*_*q*_. The detailed process of *l*th message passing is described in Figure 3. In addition, the entire message passing process is described in algorithm 1.

#### 4.3.1. Entity Nodes Update

To shorten the semantic gap between entities and the natural language question, we concatenate each node representation *e*_*m*_, node *m* ∈ *G*_*c*_, with the question node embedding *e*_*q*_, which is defined as *h*_*m*_^0^=[*e*_*m*_; *e*_*q*_]. Every time an entity node representation is updated, some new information needs to be added on the basis of the original entity embedding. This information is aggregated from the entity neighbors related to the query of the current node. In addition, our model borrows the core idea of graph attention networks [35], learns the relative weights between two connected nodes through the attention mechanism, which makes the information added from different neighbors have different weights. The difference is that in order to better adapt to the multi-hop path reasoning task, using the similarity between the relation and the question to calculate weight, instead of using the information of two adjacent nodes. Thus, in the *l*-hop graph updating stage, the representation *h*_*m*_^(*l*)^ ∈ *R*^*d*^ of each node *m* ∈ *G*_*c*_ can be updated by

(3) $$\begin{array}{c} h_{m}^{\left(l\right)}=FFN\left(h_{m}^{\left(l-1\right)},\underset{r}{\sum }\underset{k\in N_{r}\left(m\right)}{\sum }\alpha_{r}^{mk}\phi_{r}\left(h_{k}^{\left(l-1\right)}\right)\right)+h_{m}^{\left(l-1\right)}\text{,} \end{array}$$

where *FFN*( ) represents a single-layer feed-forward network, *ϕ*_*r*_( ) denotes the relation *r* specific message transformation function, and *α*_*r*_^*mk*^ is an attention weight that contains messages from node *k* to *m* connected with relation *r*.

Specifically, the attention weight *α*_*r*_^*mk*^ is the relevance probability of the query and predicate embeddings,

(4) $$\begin{array}{c} \alpha_{r}^{mk}=softmax{\left(\left(x_{r}^{\left(l-1\right)}\right.\right)}^{T}\left.h_{q}^{\left(l-1\right)}\right)\text{,} \end{array}$$

where *h*_*q*_ is the query node representation (described in equation (8) (Feq6)) and softmax( ) is the softmax normalization over all outgoing edges from node *k*. From both (3) and (4), it is observed that the current node's updated information comes more from these nodes connecting to the edges that are more relevant to that query.

As *G*_*q*_ is a multi-relational graph, the message passed from a source node to the target node should capture their relationship. Thus, the message transformation function *ϕ*_*r*_( ) calculates the information transferred from neighbor node *k* to *m*, which contains information of the edge between two nodes by introducing the relation embedding *x*_*r*_,

(5) $$\begin{array}{c} \phi_{r}\left(h_{k}^{\left(l-1\right)}\right)=M_{k}^{\left(l-1\right)}FFN\left(x_{r}^{\left(l-1\right)},h_{k}^{\left(l-1\right)}\right)\text{,} \end{array}$$

where *M*_*k*_^(*l* − 1)^ is a directed propagation matrix inspired from [12]. Combining (3) and (5), we can see that the edge information is fused into entity representation. Specifically, the directed propagation matrix uses the relevance of the query and predicates to control information flow direction,

(6) $$\begin{array}{c} M_{m}^{\left(0\right)}=\left\{\begin{array}{cc} 1\text{,} & ifm=q\text{,}\\ 0\text{,} & otherwise\text{,} \end{array}\right. \end{array}$$

(7) $$\begin{array}{c} M_{m}^{\left(l\right)}=\left(1-\lambda \right)M_{m}^{\left(l-1\right)}+\lambda \underset{r}{\sum }\underset{k\in N_{r}\left(m\right)}{\sum }\alpha_{r}^{mk}M_{k}^{\left(l-1\right)}\text{,} \end{array}$$

where (6) means that propagation starts from the query node. It can be observed from both (6) and (7) that *M* can be regard as a weight factor that controls information flow along the edge related to the query.

#### 4.3.2. Query Node Update

The initial representation of the query node is denoted as *h*_*q*_^(0)^, *h*_*q*_^(0)^=[*e*_*q*_; *e*_*q*_], similar to the other node initial representation in the graph *G*_*q*_. In *l*-layers, considering that the query node is directly connected to the topic entity node, the query representation also adds messages from the topic entity after using (3) to update with other entity nodes simultaneously,

(8) $$\begin{array}{c} h_{q}^{\left(l\right)}=FFN\left(h_{q}^{\left(l\right)},h_{s_{1}}^{\left(l\right)}\right)+h_{q}^{\left(l-1\right)}\text{,} \end{array}$$

where *h*_*s*_1__ is the topic entity representation.

#### 4.3.3. Predicate Edges Update

To obtain question-aware relation representation, during the *l*-layer graph updating process, the predicate vector connecting node *m* and *k* is updated by

(9) $$\begin{array}{c} x_{r}^{\left(l\right)}=FFN\left(x_{r}^{\left(l-1\right)},\alpha_{r}^{mk}h_{q}^{\left(l\right)}\right)+x_{r}^{\left(l-1\right)}\text{,} \end{array}$$

where *α*_*r*_^*mk*^, the similarity between the relation *r* and question *Q*, has been calculated by using (4). Residual connections are used when updating each node and edge because it can stitch together features at different levels to increase feature diversity and speed up training.

### 4.4. Answer Prediction and Training

After *L*-hop information propagation, we have final query representation *h*_*q*_^(*L*)^ and entity representation *h*_*m*_^(*L*)^ for entity *m*. The probability of this entity being the answer is calculated by the relevance score of the query and the entity representations,

(10) $$\begin{array}{c} p_{m}=\sigma {\left(\left(h_{q}^{\left(L\right)}\right.\right)}^{T}\left.h_{m}^{\left(L\right)}\right)\text{.} \end{array}$$

Locating the answers among the candidate entities in the query graph can be regarded as a node classification task, judging whether an entity node is the answer entity or not. Thus, the training process uses binary cross-entropy loss over above probabilities, which is defined as

(11) $$\begin{array}{c} L\left(\theta \right)=-\overset{n_{e}}{\underset{m=1}{\sum }}\left[y_{m}\log\right.\left(p_{m}\right)+\left(1-y_{m}\right)\log\left.\left(1-p_{m}\right)\right]\text{,} \end{array}$$

where *θ* represents the model parameters and *y*_*m*_ is the golden probability distribution over the entity.

At the testing stage, the entity with the highest score on the query graph is selected as the answer to calculate the Hit@1 metric. In addition, if the difference between the scores of other entities and the highest score does not exceed the threshold 0.1, these entities are also used as the answer selected by the model to calculate the F1 score.

### 4.5. Computation Complexity

We analyze the time and space complexity of our method and compare with prior works, GRAFT-Net [12], MHGRN [16], and QA-GNN [15] in Table 1. As we handle edges of different relation types using different edge embeddings instead of designing independent graph networks for each relation as in MHGRN, the time complexity of our method is constant with respect to the number of relations and linear with respect to the number of nodes. In addition, our model achieves the same space complexity as other models.

## 5. Experiments

### 5.1. Datasets

We used two benchmark datasets to evaluate our proposed edge-aware GNN model: MetaQA and PQL. The statistics of these datasets are described in Table 2.

MetaQA is a large-scale multi-answer dataset for KBQA in the movie domain. It contains three versions of questions, namely, Vanilla, NTM, and Audio, and each version consists of 1-hop questions, 2-hop questions, and 3-hop questions. The data form is a question-answer pair, namely, each question is followed by a list of answer entities. The dataset also provides a background KB, which contains 40128 entities and 9 relations. To make a fair comparison with previous work, we use the Vanilla version and query the given KB to predict answer for three sets of different hops.

PQL is a single-answer multi-hop KBQA dataset, which is a more challenging version in PathQuestion. The dataset consists of 2-Hop (PQL-2H) questions and 3-Hop (PQL-3H) questions, which contains 1594 and 1031 data samples, respectively. The data form is a question labeled with the golden reasoning path starting from the topic entity to the answer entity. It also provides corresponding background KB, which contains 5035 entities and 364 relations. The original dataset does not have a standard training set, test set, and dev set, we divide them at a ratio of 8 : 1 : 1 to make fair comparisons.

### 5.2. Implementation Details

#### 5.2.1. Experimental Settings

We run the experiments on a V100 GPU with 16G memory. The batch size is set to 32. All the embeddings are initialized randomly. The hidden dimension of the LSTM is 300. The hidden dimension of all GNN layers is set to 300. The layer number is 4 for all GNNs in 2-hop settings and 5 in 3-hop settings. The dropout rate is set to 0.2. The Adam optimizer [50] is used with the learning rate of 0.001.

#### 5.2.2. Data Pre-Processing

First, entity linking is performed to get the topic entity of a question. For entity linking, we use simple surface level matching. Then, query the background KB to obtain entities and predicates within *n* hops for a *n*-hop question and obtain a question-related subgraph. For the PQL dataset, all entities and predicates within *n* hops for a *n*-hop question are kept to construct the subgraph. For the MetaQA dataset, the maximum number of fact triples retrieved for a question is very large. To fit into GPU memory for gradient-based learning, the size of the retrieved subgraph is limited. We randomly remove some non-answer entities and predicates from the obtained *n*-hop subgraph. The statistics of the final subgraph input to the model are shown in Tables 3 and 4, respectively.

### 5.3. Baselines

We compare our model with the following baselines:

KV-MemNN: It was proposed by the authors of [51], which is an end-to-end memory network reasoning on the key-value structured memory storing KB facts. This model learns to use keys storing the subject and predicate to address relevant memories with respect to the question, whose corresponding values storing the object are subsequently returned.

IRN: It was proposed by the authors of [18], which is an interpretable hop-by-hop reasoning network. In each hop of reasoning, the model dynamically predicts a relation according to the corresponding part of the input question, and updates the state of both the reasoning process and the question representation utilizing the predicted relation.

VRN: It was proposed by the authors of [17], which is an end-to-end variational reasoning network to recognize the topic entity of the input question and learn multi-hop reasoning simultaneously in a unified probabilistic framework. In terms of logic reasoning task, the model uses a propagation-like deep learning architecture over the KB.

GRAFT-Net: It was proposed by the authors of [12], which is a graph convolution based neural network performing question answering over the combination of a KB and entity-linked text. The model uses a novel update rule to operate over heterogeneous graphs and a directed propagation method to constrain the reasoning starting from the topic entity.

SGReader: It was proposed by the authors of [47], which combines the unstructured text and KB triples to predict answers, where the SGReader employs graph attention networks to accumulate information for each entity in the question-related subgraph and the KAReader utilizes a gating mechanism to selectively incorporate the learned entity information into encoding the question and texts.

2HR-DR: It was proposed by the authors of [2], which is a directed hypergraph convolutional network-based model. The model learns the relation representation by connected entity features, allocates the weight dynamically for different relations, and then updates the entity representation based on dynamic relation weights.

GlobalGraph: It was proposed by the authors of [14], which is a GNN-based model capturing long-distance node relations by modeling the relation features of each node and further judging the feature similarity.

For KV-MenNN, GraftNet, and SGreader, the experiment results on MetaQA and PQL datasets are provided by [14].

### 5.4. Main Results and Analysis

Following the work proposed by Wang et al. [14], we employ the Hits@1 and F1 score to measure the performance of the models for the MetaQA dataset, and adopt Hits@1 for evaluating the PQL dataset.

Table 5 demonstrates the performance of the baseline methods and our model on the MetaQA dataset. Our model outperforms all baselines on the MetaQA 2-Hop and MetaQA 3-Hop dataset, improving Hits@1/F1 by 1.3%/10.7% and 14.9%/28.6%, respectively. In addition, for MetaQA 1-Hop, we obtain competitive Hits@1 and improve F1 from 97.6% to 98.5%. This reason for the relatively low Hits@1 on MetaQA 1-Hop is that models like GlobalGraph use the PageRank algorithm to pre-prune some candidate entities, but our model does not use any prior knowledge in data pre-processing. In general, our model makes a great improvement on the F1 score, which means our model achieves a higher recall while ensuring precision. This is because relation information is added to the message passing process so that the model gives similar scores to the entity nodes that arrive on the same relation path, thereby identifying a series of answer entities and improving the recall rate. Besides, our model performs better on multi-hop questions than 1-hop questions because of the reasoning advantage of graph propagation in dealing with multi-hop questions.

As shown in Table 6, our method achieves the best Hits@1 compared with the baseline models on the PQL 2-Hop dataset, which remains a great improvement, 9.6% higher than the second best model. It also obtains a good result on PQL-3H, 1.0% higher than the third best one and 1.0% lower than the best one. Note that the original PQL dataset does not provide a standardized training, test, and dev set; therefore, the way that the dataset is divided greatly affects the experimental results. Because the data in this dataset has many duplicates, if the test set contains data that is similar to the train set, the experimental result will be very high. Thus, we have adopted five division methods to avoid similar data in the test set and the train set as much as possible. The experiments are repeated 5 times, and the average value and fluctuation range in the table were obtained. Combined with the fluctuation range, our experimental results are still quite competitive.

### 5.5. Performance Analysis

#### 5.5.1. Ablation Study on Model Components

We conduct ablation experiments to evaluate the performance of different components in our model, and the experimental results illustrate the effectiveness of these components. Note that w/o predicate edges update does not consider updating the predicate information represented by the edges in the query graph, which only performs nodes update. w/o query node update does not consider updating query node representation. w/o interaction between query and predicates removes similarity between query and predicates as the propagation weight and performs information propagation based on the neighbors of nodes. The w/o query node does not consider constructing the query graph but uses the candidate entity graph. As shown in Table 7, we can find that our overall model achieves the best performance. Without these components, the performance of the model has declined, which demonstrates the effectiveness of the design of graph construction and update in our model. Specially, by comparing w/o interaction between query and predicates and w/o predicate edges update, the results illustrate the significance of relation information, which could guide the model to choose the best matching path with the question hop by hop.  Table 8 shows some case studies to analyze our model's behavior. Using our full model can better answer a major category of questions, that is, questions that contain loops, which means there are repeated triples in the reasoning path, such as the first and third examples. In addition, through these examples, it can be observed that the reasoning path related to the question cannot be obtained without predicate updating or interaction components, confirming the importance of relation information.

#### 5.5.2. Impact of Number of Hops (L)

We investigate the impact of hyperparameter *L* for the edge-aware GNN with experiments on MetaQA 1-Hop (Figure 4). The increase of *L* continues to bring benefits until *L*=3. Performance begins to drop when *L* > 3, which might be attributed to the noise caused by longer relation paths in the knowledge base. However, deep hops will not greatly affect the experimental effectiveness. We believe that this is because the addition of the query node enables the question information to be better integrated into other entity nodes and relation edges, thereby reducing the introduction of irrelevant information in the process of deep message passing.

## 6. Conclusion and Future Work

Multi-hop path reasoning over knowledge base aims to find the answer entities in graphical data that contains rich relation information among entities. In this paper, we proposed an edge-aware GNN model to deal with this kind of graph. Our model first adopts a special graph construction way to enable smooth information interaction between the question and the candidates. Then, it updates the vector representation of each element in the graph by introducing question-related relation information. Finally, the edge-aware GNN model predicts the answers by calculating the correlation between the question and node entities. Experiments on the MetaQA and PQL benchmarks demonstrate that the proposed model achieves better Hit@1 and F1 scores than the state-of-the-art models by a large margin. Furthermore, both the constructed query graph and the graph update algorithm contribute to the performance improvement.

This work opens several interesting directions for future research. First, the proposed GNN-based model can be well applied to single or multi-hop questions. We can further explore the application of GNN in reasoning questions with constraints such as aggregation and comparison in the following work. In addition, this paper focuses on answering questions that contain only one topic entity. If there are multiple topic entities in the question or the topic entity is not clear, we will treat this fuzzy phenomenon as future work.

## Figures and Tables

**Figure 1:** A concrete example of multi-hop path reasoning over the knowledge base. Given a “*what type*” question, we aim to derive the answer (black red oval box) by following the corresponding multi-hop triplet path (red font) starting from the topic entity (yellow oval box) in the graph.

**Figure 2:** Overview of our approach. Given a question, we retrieve relevant entities from a KB to obtain candidate graph, connect the question with the retrieved graph to form a query graph (§4.1), initialize both the node and edge representation on the graph (§4.2), update graph nodes and edges (§4.3), and predict the answer (§4.4).

**Figure 3:** During *l*-hop graph updating, the entity node update takes *s*_1_ as an example, and the relation edge update takes *r*_*q*_ as an example. It should be noted that all nodes and edges will be updated at each hop. For ease of drawing, the update operation of non-query nodes is described separately. The left side describes the entity node representation *h*_*s*_1__ update process, and the right side describes the question node representation *h*_*q*_ and edge representation *x*_*rq*_ update process.

**Figure 4:** Effect of (L) in the edge-aware GNN. We show Hits@1 on MetaQA 1-Hop with respect to hops.

**Algorithm 1:** Multi-hop edge-aware message passing algorithm.

**Table 1:** Computation complexity of different L-hop question answering models on a graph *G*={*𝒱*, *ℰ*, *ℛ*}.

Model	Time	Space
L-hop GRAFT-Net	*𝒪*(|*ℛ*‖*𝒱*|*L*)	*𝒪*(|*ℛ*‖*𝒱*|*L*)
L-hop MHGRN	*𝒪*(|*ℛ*|^2^|*𝒱*|^2^*L*)	*𝒪*(|*ℛ*‖*𝒱*|*L*)
L-hop QA-GNN	*𝒪*(|*𝒱*|^2^*L*)	*𝒪*(|*ℛ*‖*𝒱*|*L*)
L-hop ours	*𝒪*(|*ℛ*‖*𝒱*|*L*)	*𝒪*(|*ℛ*‖*𝒱*|*L*)

**Table 2:** The statistics of the datasets.

Datasets		Train	Valid	Test	Entities	Relations
MetaQA	1-Hop	96106	9992	9947	40128	9
	2-Hop	118980	14872	14872		
	3-Hop	114196	14274	14274		

PQL	2-Hop	1274	160	160	5035	364
	3-Hop	925	103	103		

**Table 3:** The statistics of the subgraph input to the model on PQL.

	PQL 2-hop	PQL 3-hop
	Train || test || dev	Train || test || dev
max facts	416 || 416 || 184	1704 || 1508 || 250
max entities	204 || 204 || 92	852 || 755 || 125
avg. Entities	19.77 || 18.01 || 19.61	36.30 || 27.06 || 17.97

**Table 4:** The statistics of the subgraph input to the model on MetaQA.

	MetaQA 1-hop	MetaQA 2-hop	MetaQA 3-hop
	Train || test || dev	Train || test || dev	Train || test || dev
max facts	230 || 204 || 204	780 || 754 || 776	742 || 732 || 728
max entities	102 || 102 || 102	253 || 195 || 245	264 || 264 || 266
avg. Entities	9.26 || 9.31 || 9.15	32.19 || 32.07 || 32.52	137.93 || 136.96 || 137.64

**Table 5:** Experimental results on the MetaQA dataset.

Model	MetaQA 1-hop		MetaQA 2-hop		MetaQA 3-hop	
	Hits@1	F1	Hits@1	F1	Hits@1	F1
KV-MemNN	0.958	—	0.760	—	0.489	—
VRN	0.975	—	0.899	—	0.625	—
SGReader	0.967	0.960	0.807	0.798	0.610	0.580
GRAFT-Net	0.974	0.910	0.948	0.727	0.778	0.561
2HR-DR	0.988	0.973	0.937	0.814	—	—
GlobalGraph	**0.990**	0.976	0.955	0.830	0.814	0.624
Ours	0.972	**0.985**	**0.968**	**0.937**	**0.963**	**0.910**

The best results are indicated in bold values.

**Table 6:** Experimental results on the PQL dataset.

Model	PQL 2-hop	PQL 3-hop
	Hits@1	Hits@1
KV-MemNN	0.622	0.674
IRN	0.725	0.710
SGReader	0.719	0.893
GRAFT-Net	0.707	0.913
2HR-DR	0.755	0.921
GlobalGraph	0.760	**0.941**
Ours	**0.856**(±0.050)	0.931(±0.019)

The best results are indicated in bold values.

**Table 7:** Ablation experiments of our model on the PQL dataset.

Model	PQL 2-hop	PQL 3-hop
	Hits@1	Hits@1
Ours	0.856	0.931
w/o predicate edges update	0.813 (−4.3%)	0.850 (−8.1%)
w/o query node update	0.825 (−3.1%)	0.890 (−4.1%)
w/o interaction between query and predicates	0.800 (−5.6%)	0.879 (−5.2%)
w/o query node	0.838 (−1.8%)	0.906 (−2.5%)

**Table 8:** Case studies from the PQL 3-Hop dataset, comparing prediction results by our total model (ours), w/o predicate edges update (w/o PU), w/o query node update (w/o QU), w/o interaction between query and predicates (w/o Intr), and w/o query node (w/o QN).

Question (golden reasoning path)	Ours	w/o PU	w/o Qu	w/o intr	w/o Qn
What is the notable types of release of Free's release? (Free, music_release,Free, music_release,Free, notable_types, Consumer product)	Consumer product (√)	Free (×)	Free (×)	Free (×)	Free (×)

What is the author of tracks of Reminiscense's track list? (Reminiscense, music_tracklist,Evolution, music_tracks,Evolution, book_author, Charles Darwin)	Charles Darwin (√)	Evolution (×)	Musical Album (×)	Evolution (×)	Charles Darwin (√)

What is the artist of releases of new Orlean's releases? (New Orlean, music_releases, New Orlean, music_releases, New Orlean, music_artist, Idris Muhammad)	Idris Muhammad (√)	Web development (×)	Idris Muhammad (√)	Web development (×)	Idris Muhammad (√)

What is the place of birth of people born here of Thomas Joseph Drury's place of birth? (Thomas Joseph Drury, place_of_birth,Ballymote, people_born_here, Thomas Joseph Drury, place_of_birth,Ballymote)	Ballymote (√)	Ballymote (√)	Thomas Joseph Drury (×)	Ballymote (√)	Brother Walfrid (×)

What is the release type of recording of Cold War's recording? (Cold War,music_recording, Cold War,music_recording, Cold War, release_type,EP)	EP (√)	EP (√)	EP (√)	Cold War (×)	EP (√)

## Data Availability

The data used to support the findings of this study are available at https://github.com/zmtkeke/IRN and https://goo.gl/f3AmcY.
